The article "Myricetin Inhibited Fear and Anxiety-Like Behaviors by HPA Axis Regulation and Activation of the BDNF-ERK Signaling Pathway in Posttraumatic Stress Disorder Rats" was published in 2022. Journal: Evid Based Complement Alternat Med.

# Myricetin Inhibited Fear and Anxiety-Like Behaviors by HPA Axis Regulation and Activation of the BDNF-ERK Signaling Pathway in Posttraumatic Stress Disorder Rats

**DOI:** 10.1155/2022/8320256

**Published:** 2022-06-08

**Authors:** Bongjun Sur, Bombi Lee

**Affiliations:** Acupuncture and Meridian Science Research Center, Kyung Hee University, Seoul, Republic of Korea

## Abstract

Posttraumatic stress disorder (PTSD) is a stress-related psychiatric or mental disorder characterized by experiencing a traumatic stress. The cause of such PTSD is dysregulation of the hypothalamic-pituitary-adrenal (HPA) axis and imbalance of monoamines. Myricetin (MYR) is a common natural flavonoid that has various pharmacological activities. We investigated the effects of MYR on fear, depression, and anxiety following monoamine imbalance and hyperactivation of HPA axis in rats exposed to a single prolonged stress (SPS). Male rats were dosed with MYR (10 and 20 mg/kg, i.p.) once daily for 14 days after exposure to SPS. Administration of MYR reduced freezing responses to extinction recall, depression, and anxiety-like behaviors and decreased increase of plasma corticosterone and adrenocorticotropic hormone levels. Also, administration of MYR restored decreased serotonin and increased norepinephrine in the fear circuit regions, medial prefrontal cortex, and hippocampus. It also increased the reduction in the brain-derived neurotrophic factor (BDNF) and tropomyosin-related kinase B mRNA expression and the ratio of p-ERK/extracellular signal-regulated kinase (ERK) in the hippocampus. Thus, MYR exerted antidepressant and anxiolytic effects by regulation of HPA axis and activation of the BDNF-ERK signaling pathway. Finally, we suggest that MYR could be a useful therapeutic agent to prevent traumatic stress such as PTSD.

## 1. Introduction

Post-traumatic stress disorder (PTSD) is a serious psychological disorder that affects people who have experienced unexpected or traumatic events, such as sexual assault, a natural disaster, or war, or even exposure to disaster-related news [1, 2]. Furthermore, more than 70% of the world's population will be exposed to at least one traumatic event in their lifetime and more than 17% will be diagnosed with PTSD [3]. PTSD is characterized by re-experience, avoidance, and hyperarousal [4, 5]. Chronic PTSD is also associated with other psychiatric disorders, such as anxiety, depression, drug addiction, sleep disturbances, and memory impairment [6, 7]. Given its associated psychological and occupational impairments, PTSD is emerging as a social problem [4].

Neurobiological factors implicated in PTSD include activation of the monoamine system, changes in the neuroendocrine system, and dysregulation of the hypothalamic-pituitary-adrenal (HPA) axis [8–10]. In other words, it is caused by traumatic stress-induced emotional fear memory and anxiety-like symptoms, arising through an imbalance among neurotransmitters, such as serotonin (5-HT), dopamine, and norepinephrine (NE), in the fear circuit regions (e.g., the medial prefrontal cortex (PFC), hippocampus (HIP), and amygdala (AMY)) [11]. Decreased 5-HT and increased NE were observed in the PFC and HIP of PTSD patients [9]. PTSD patients also maintain high concentrations of glucocorticoids (GCs) because of HPA axis, dysregulation and stress amplification caused by increased adrenocorticotropic hormone (ACTH), corticotropin-releasing hormone (CRH), and NE activity [12]. Human and animal studies have demonstrated increased circulating GC levels as a result of exposure to excessive stress, leading to overactivation of the AMY and impaired extinction of fear learning [13, 14].

Several studies have also reported that stress-induced elevation of corticosterone (CORT) increased the fear response by decreasing the expression of brain-derived neurotrophic factor (BDNF) and its receptor, tropomyosin-related kinase B (TrkB) [15, 16].

Selective serotonin reuptake inhibitors (SSRIs) and serotonin and norepinephrine reuptake inhibitors (SNRIs), which are currently used as therapeutic agents for PTSD, have limited effectiveness and cause various side effects, such as withdrawal, sedation, dependence, and cognitive dysfunction [17, 18]. Therefore, there is a need for new safe and effective drugs.

Myricetin (MYR; 3,3′,4′5,5′,7-hexahydroxylflavone) is a natural flavonoid found in berries, vegetables, teas, and the fruits of various plants [19]. MYR has various pharmacological effects, including antioxidant, antiapoptotic, anti-photoaging, anticancer, antidiabetic, and anti-inflammatory effects [20–24]. In particular, MYR showed neuroprotective effects in the HIP of stressed mice and reduced neuronal damage in animal models of neurodegenerative diseases (e.g., ischemic stroke, epilepsy, Parkinson's disease, and Alzheimer's disease) [25–27]. MYR attenuated brain damage in a rat model of cerebral ischemia by activating the nuclear factor (erythroid-derived 2)-like 2 pathway and reducing oxidative stress [28]. A growing body of evidence suggests the potential of MYR as a therapeutic option for preventing stress- and trauma-related psychiatric conditions, including PTSD.

In this study, a single prolonged stress (SPS) was used to induce PTSD-like symptoms in an animal model, through recall of fear extinction [29]. This model is based on the finding that people with multiple or early traumas are more likely to develop PTSD after a traumatic event [30].

We evaluated the effects of MYR on depression- and anxiety-like behaviors in rats exposed to SPS using the fear conditioning test (FCT), forced swim test (FST), and elevated plus maze (EPM) test. Moreover, we investigated regulation of the HPA axis and neurotransmitters and activation of the BDNF-extracellular signal-regulated kinase (ERK) signaling pathway, which leads to stress-induced behavioral alterations.

## 2. Methods

### 2.1. Animals and MYR Administration

As experimental animals, 6- to 7-week-old male Sprague-Dawley rats (200∼220 g; Samtaco Animal Co., Seoul, Korea) were used. All animal care and experimental procedures were conducted in accordance with the National Institute of Health Guide for the Care and Use of Laboratory Animals and were approved by the Kyung Hee University Institutional Animal Care and Use Committee (KHUASP(SE)-21-045).

The rats were divided into five groups: saline-treated normal control (SAL) group, SPS only group, MYR treatment groups, and positive control (PAX) group (*n* = 8/groups). For the experiment, the standard doses of MYR (10 and 20 mg/kg, Sigma-Aldrich Chemical Co., St. Louis, MO, USA) and paroxetine hydrochloride (15 mg/kg, PAX, positive control; Sigma-Aldrich) were determined based on a previous study [25]. MYR and PAX were dissolved in 0.9% saline before use and were injected intraperitoneally (i.p.) once daily for 14 days. The experimental schedule is shown in Figure 1.

### 2.2. SPS

In the SPS animal model, rats were immobilized for 2 hours, forced to swim for 20 min, and then rested for 15 min. After rest, rats were exposed to isoflurane (2–3%) until losing consciousness. For sensitization, rats were left alone in cages for 7 days [31].

### 2.3. Behavioral Test

To evaluate the fear response (FCT), rats were acclimatized to a fear conditioned box (30 cm × 30 cm × 30 cm). On day 1, rats were initiated the conditioning trials for 1 min in the box. When a rat entered the box, a conditional stimulus (sound alarm: 30 sec, 85 dB) was applied. For fear stimulation, during the last 2 sec of the conditional stimulus, a single electric footshock (0.5 mA, 2 sec) was applied (as an unconditional stimulus, forming the learning trial). On day 2, when the rats entered the box from a railing, no conditional stimuli or shocks were applied, forming the extinction training. After 24 hours, for extinction recall, the rats were re-exposed to the conditional stimulus alone in the same chamber without any electric footshock, and we observed the rat's fear response for 5 min. The fear response was the duration of the freezing response with no movement other than breathing.

To evaluate the depression-like behavior (FST), rats were forced to swim in a water bath (20 cm diameter × 50 cm height) filled to a depth of 30 cm with 25°C water for 5 min. Rats that did not swim and were floating were considered to be in a depressed state (immobility), as described previously [31].

To evaluate anxiety-like behavior using the apparatus detailed in a previous study (EPM test) [32], rats were placed in the center of a maze and tested for 5 min. The apparatus consisted of two open arms (50 cm × 10 cm) and two closed arms with dark walls (50 cm × 10 cm × 50 cm). The maze was 50 cm above the ground and the arms were connected by a platform (10 × 10 cm). The time spent in and number of visits to the two open and two closed arms were measured. Behavior in the maze was measured by the S-MART program (PanLab, Barcelona, Spain).

Also, in the sucrose preference test, intake of water and sucrose solution (1%, w/v) was measured for 3 h, as described previously [31].

### 2.4. Enzyme-Linked Immunosorbent Assay to Assess Neurotransmitter Levels

Plasma levels of CORT (Novus Biologicals, LLC., Littleton, CO, USA), ACTH (Abcam, Cambridge, UK), and CRH (Biocompare, South San Francisco, CA, USA) and concentrations of 5-HT (Abcam) and NE (Novus Biologicals) in the PFC, HIP, and AMY were measured by competitive enzyme-linked immunosorbent assay (ELISA), as described previously [31]. Each group (*n* = 4/groups) was anesthetized through inhalation of isoflurane (2%; Hanlim Pharm., Seoul, Korea) for 5 to 10 seconds in random order and was killed by sacrifice one day after the behavioral testing. Plasma was collected via the abdominal aorta (*n* = 4/groups), after which the PFC, HIP, and AMY were quickly dissected from the rat brains.

### 2.5. Immunohistochemistry

Immunohistochemistry was also performed to evaluate the number of BDNF-immunoreactive neurons in the HIP, as described previously [31]. The rats (*n* = 4/groups) were deeply anesthetized with sodium pentobarbital (80 mg/kg, by intraperitoneal injection) and perfused through the ascending aorta with normal saline (0.9%), followed by 300 ml (per rat) of 4% paraformaldehyde in 0.1 M phosphate-buffered saline (PBS). The brains were removed, postfixed overnight, and cryoprotected with 20% sucrose in 0.1 M PBS at 4°C. Coronal sections of 30 *μ*m thick were cut through the HIP using a cryostat (Leica CM1850; Leica Microsystems Ltd., Nussloch, Germany). The tissue sections were obtained according to the rat Atlas of Paxinos and Watson (HIP; between bregma −2.6 and −3.6) [33]. The tissue sections were incubated overnight with primary rabbit anti-BDNF antibody (1 : 200 dilution, Cell Signaling, Boston, MA, USA), and the sections were then incubated for 2 hours at room temperature with secondary antibodies (1 : 200 dilution; Vector Laboratories Co., Burlingame, CA, USA). Next, the sections were incubated with avidin-biotin-peroxidase complex (Vector Laboratories) for 1 hour at room temperature and then in a solution containing 3,3′-diaminobenzidine (DAB; Sigma-Aldrich) and 0.03% hydrogen peroxide for 1 min. Images were captured using the AxioVision 3.0 imaging system (Carl Zeiss, Inc., Oberkochen, Germany) and processed using Adobe Photoshop (Adobe Systems, Inc., San Jose, CA, USA). The sections were viewed at 200x magnification, and the numbers of cells within 100 × 100 mm^2^ grids were counted by observers blinded to the experimental groups. Hippocampal area cells were obtained according to the stereotactic Atlas of Paxinos and Watson [33]. The cells were counted in three sections per rat within the hippocampal area.

### 2.6. Total RNA Preparation and Reverse Transcription-Polymerase Chain Reaction

TRIzol reagent (Sigma-Aldrich) was added to the HIP isolated from the brain to recover the total RNA. After cDNA was synthesized from RNA by reverse transcription reaction, polymerase chain reaction (PCR) was performed as described previously [31]. The PCR products were separated on 1.2% agarose gel and stained with ethidium bromide after which the density of each band was evaluated using an image-analyzing system (i-Max™; CoreBio System Co., Seoul, Korea). Complementary DNA expression levels were determined by calculating the relative density of each BDNF and TrkB bands to GAPDH.

### 2.7. Western Blot Analysis

Total protein was extracted from the brain to detect ERK protein in the HIP. To extract total protein, brain tissue was homogenized with lysis buffer containing a phosphatase inhibitor and a protease inhibitor (CyQUANT; Invitrogen, Carlsbad, CA, USA). To separate proteins from the homogenized sample, the supernatant was collected by centrifugation (12,000 rpm, 15 min, 4°C). The protein concentration was measured using a colorimetric protein assay kit (Bio-Rad, Hercules, CA, USA). Protein samples (15–20 *µ*g) were resolved using 10% sodium dodecyl sulfate-polyacrylamide gel electrophoresis at 120 V and then electrotransferred to a nitrocellulose membrane (Schleicher and Schuell GmbH, Dassel, Germany). After incubation with a mouse p-ERK antibody (1 : 500; Cell Signaling, Danvers, MA, USA), the membrane was incubated with horseradish peroxidase conjugated goat anti-mouse IgG secondary antibody (Santa Cruz Biotech, Santa Cruz, CA, USA). A chemiluminescent kit (Super Signal West Pico; Pierce, Rockford, IL, USA) was used to detect the p-ERK protein. Protein content was analyzed using an enhanced chemiluminescence detection system (Santa Cruz), and the density was measured using the Tina 2.1 program.

### 2.8. Statistical Analysis

Data are presented as the mean ± standard error. To test for statistical differences between groups, all data were analyzed using SPSS software (version 23.0; SPSS, Inc., Chicago, IL, USA). Data sets were checked for normality and homogeneity of variances by Shapiro–Wilk and Brown–Forsythe tests, respectively. One-way ANOVA followed by Tukey's *post hoc* test or Kruskal–Wallis test with Dunn's multiple comparison *post hoc* test was used to compare multiple comparisons such as the behavioral test, ELISA, PCR, western blot, and immunohistochemistry analysis. *p* < 0.05 was considered statistically significant.

## 3. Results

### 3.1. Effect of Body Weight and Sucrose Intake according to SPS

Rats exposed to SPS showed a significant decrease in the change of body weight over time compared to the saline-treated normal (SAL) group (*t* = 4.724, *p* < 0.01). This change in body weight showed a significant difference from day 3 after exposure to SPS (Figure 2(a)).

Rats exposed to SPS showed a significant decrease in sucrose intake on days 7 and 14 compared to the SAL group (*t* = 869, *p* < 0.01; Figure 2(b)). The rats exhibited sufficient physiological changes and anhedonia due to traumatic stress following SPS exposure.

### 3.2. Effect of MYR in Behavioral Changes by SPS

In the FCT, the rats exposed to SPS showed a similar pattern of freezing responses to the fear stimulus (conditioning trials, C1–C3) compared to the SAL group (*t* = 0.254, *p* = 0.808; Figure 3(a)). During fear stimulus in both extinction (E1–E6) and extinction recall (R1; short-term recall), the rats exposed to SPS showed a significantly increased freezing response compared to the SAL group (*p* < 0.01 and *p* < 0.001, respectively). However, administration of 20 mg/kg MYR significantly decreased the freezing response during extinction recall compared to the SPS group (*p* < 0.05; Figure 3(b)), indicating that the freezing response of the MYR20 group was similar to that of the PAX group.

In the FST, the rats exposed to SPS had a significantly increased immobility time and decreased climbing time compared to the SAL group (*p* < 0.01; Figures 3(c) and 3(d)). Administration of 20 mg/kg MYR significantly decreased the immobility time (*p* < 0.05) and increased the climbing time (*p* < 0.05) compared to the SPS group. Similarly, rats in the PAX group decreased immobility time in the FST, but it was not statistically significant (*p* = 0.078, Figure 3(c)). Also, there was no difference in swimming time among all groups (*F*_4,34_ = 0.245, *p* = 0.910; Figure 3(e)).

In the EPM test, the percentage of time spent in and the number of entries into the open arms of rats exposed to SPS was significantly decreased compared to the SAL group (*p* < 0.01; Figures 3(f) and 3(h)). However, administration of 20 mg/kg MYR significantly increased the percentage of time spent in and the number of entries into the open arms compared to the SPS group (*p* < 0.05). Our results show that increase in the percentage of time spent in the open arms in the MYR20 group was comparable to the exploratory behavior. Similarly, the rats in the PAX group had significantly increased the percentage of time spent in the open arms of the maze (*p* < 0.05). Among all the groups, the time spent in and the number of entries into and in the closed arms did not differ (*F*_4,34_ = 0.900, *p* = 0.476 and *F*_4,34_ = 2.477, *p* = 0.065, respectively; Figures 3(g) and 3(i)). Administration of 20 mg/kg MYR significantly decreased the anxiety index compared to the SPS group (*p* < 0.05; Figure 3(j)), indicating that the anxiety-like behaviors of the MYR20 group were similar to those of the PAX group.

### 3.3. Effect of MYR in HPA Axis Activation and Neurotransmitters Changes by SPS

Rats exposed to SPS had significantly increased plasma CORT level compared to the SAL group (*p* < 0.01; Figure 4(a)). Compared to the SAL group, the rats exposed to SPS had significantly increased plasma ACTH level (*p* < 0.01; Figure 4(b)), but there was no significant difference in plasma CRH level (*p* = 0.995; Figure 4(c)). However, the administration of 20 mg/kg MYR significantly decreased the plasma CORT and ACTH levels compared to the SPS group (*p* < 0.05). Similarly, rats in the PAX group had significantly decreased the plasma CORT level compared to the SPS group (*p* < 0.05).

Rats exposed to SPS had significantly increased NE concentrations in the PFC, HIP, and AMY compared to the SAL group (*p* < 0.05 and *p* < 0.01, respectively; Figures 4(d)–4(f)). The administration of 20 mg/kg MYR significantly decreased the NE concentrations in the HIP and AMY compared to the SPS group (*p* < 0.05). Similarly, rats in the PAX group had significantly decreased the NE concentration in the AMY compared to the SPS group (*p* < 0.05).

Rats exposed to SPS had significantly decreased 5-HT concentrations in the PFC and HIP compared to the SAL group (*p* < 0.05 and *p* < 0.01, respectively; Figures 4(g) and 4(h)), but there was no significant difference in 5-HT concentration in the AMY (*p* = 0.427; Figure 4(i)). However, the administration of 20 mg/kg MYR significantly increased the 5-HT concentrations in the PFC and HIP compared to the SPS group (*p* < 0.05). Similarly, rats in the PAX group had significantly increased the 5-HT concentration in the HIP compared to the SPS group (*p* < 0.05).

### 3.4. Effect of MYR in Immunohistochemical Changes of BDNF by SPS

In the HIP, the number of BDNF-immunopositive neuronal cells in the SPS group was significantly decreased compared to those in the SAL group (*p* < 0.05; Figure 5). The BDNF-reactive neuronal activity in the HIP was significantly increased in the hippocampal region in the MYR20 group compared to those in the SPS group (*p* < 0.05).

### 3.5. Effect of MYR in BDNF and TrkB mRNA Expression by SPS

Compared to the SAL group, SPS exhibited significantly reduced BDNF mRNA expression in the HIP (*p* < 0.01; Figure 6(a)). However, the administration of 20 mg/kg MYR significantly increased the BDNF mRNA level in the HIP compared to the SPS group (*p* < 0.05; Figure 6(a)).

Compared to the SAL group, SPS exhibited significantly reduced TrkB mRNA expression in the HIP (*p* < 0.05). However, the administration of 20 mg/kg MYR increased the TrkB mRNA level in the HIP compared to the SPS group, although this result was only marginally significant (*p* = 0.196).

### 3.6. Effect of MYR in p-ERK Activation by SPS

The effect of MYR on the protein expression level of p-ERK in hippocampal tissue were determined by Western blotting. The SPS group showed a significant decrease in p-ERK protein expression level in the HIP compared to the SAL group (*p* < 0.01; Figure 6(b)). However, the administration of 20 mg/kg MYR significantly increased the p-ERK protein expression level in the HIP compared to the SPS group (*p* < 0.05).

## 4. Discussion

In this study, the effects and possible mechanism of action of MYR on the fear response, depression, and anxiety-like behaviors induced by PTSD were evaluated using an SPS model. MYR administration after exposure to SPS significantly reduced the freezing response in the FCT, significantly increased the percentage of time spent in and the number of entries into the open arms of the EPM test, and significantly decreased immobility time in the FST. MYR administration also significantly reduced the increase in CORT and ACTH levels induced by HPA axis dysregulation and regulated the imbalance of NE and 5-HT concentrations in the fear circuit regions (PFC, HIP, and AMY). In addition, MYR treatment restored BDNF mRNA and p-ERK protein expression in the HIP. Thus, MYR relieved depression and anxiety through regulation of the HPA axis, neurotransmitters in the brain fear circuit regions, and the BDNF-ERK signaling pathway. These findings could lead to the development of a new therapeutic agent for PTSD.

SPS can induce cognitive dysfunction [34], an exaggerated startle response [35], heightened fear [36], and depressive and anxiety-like behaviors.

In this study, SPS exposure led to a decrease in the body weight and sucrose intake of rats compared to the controls. Increased anhedonia after SPS exposure in rats suggests that traumatic stress can induce depression [37]. Although body weight loss is not a direct indicator of fear, depression, or anxiety, various physiological changes are associated with SPS exposure [37].

PTSD patients are known to develop a fear response due to impairment of the extinction of traumatic memory [38, 39]. This is consistent with the hypersensitivity and increased fear circuit activation seen in PTSD patients exposed to another potentially threatening stimulus [38, 39]. Several studies have demonstrated impaired fear extinction in the passive avoidance task in SPS-exposed rats, which also exhibited enhanced anxiety responses in the EPM test [40] and light/dark box task [34] due to the reinforcement of fear memory. In our study, in agreement with previous studies, rats exposed to single electric footshocks and conditional stimuli in the FCT had a significantly increased freezing response during fear extinction (E1∼E6) and extinction recall (R1). The SPS-exposed rats did not learn to recognize a safe space or situation even when the threat was removed due to HPA-axis dysregulation and activation of the fear circuit regions (PFC and HIP) [41]. However, MYR administration alleviated the impaired fear extinction by reducing freezing behavior, followed by attenuation of fear during short-term extinction recall. Therefore, MYR administration may improve depression- and anxiety-like behaviors, as well as fear memory, by enhancing fear extinction.

Depression- and anxiety-like behaviors were comorbid symptoms in both human and animal studies of PTSD [38]. After SPS exposure, rats exhibited increased immobility time in the FST. A heightened state of fear and behavioral despair were observed following traumatic stress and forced swimming. In addition to the FST, exposure of rats to SPS in the EPM test significantly decreased the percentage of time spent in and the number of entries into the open arms. The decreased searching for the open arm reflected an increase in anxiety-like behavior due to an aversive experience, as is also seen when faced with another threatening situation [42]. These results suggested that increased depression- and anxiety-like behaviors were associated with changes in CORT and monoamine levels in various brain regions [43]. However, our results indicate that MYR administration can help restore the SPS-induced depression and anxiety-like behaviors.

Many studies have reported that the biochemical and endocrine abnormalities seen in PTSD patients are well reproduced in SPS animal models [36]. Long-term exposure to CORT has been also shown to produce neurotoxic effects in anxiety-related brain regions, such as the HIP and AMY [44]. In our study, SPS exposure increased plasma CORT and ACTH levels in rats, resulting in HPA axis dysfunction. PTSD-related HPA axis dysregulation implied impairment of important neuroendocrine systems regulating immune function, energy expenditure, emotion and mood, and stress [45]. Sustained CORT elevation may cause biochemical, metabolic, and structural changes in the HIP and AMY, leading to behavioral changes seen in PTSD, such as pathophysiological and anxiety-like behaviors [46]. However, MYR administration reduces plasma CORT and ACTH levels, spontaneous HPA axis excitability, and HPA axis dysregulation, thereby alleviating fear memory and depression- and anxiety-like behaviors.

The fear circuit of the brain is involved in fear extinction, which is an important feature of PTSD known to affect other systems related to fear extinction [47]. In PTSD patients, catecholamine imbalances occur due to disturbances in the adrenergic system in the fear circuit regions [48]. Increased NE is associated with avoidance and the re-experiencing of traumatic stress [49]. Our results also demonstrate that SPS-exposed rats had increased NE levels in the PFC, HIP, and AMY. However, MYR administration suppressed the SPS-related NE increase in HIP and AMY. This suggests that MYR administration could modulate the imbalance of catecholamines, which is a known pathophysiological cause of PTSD.

Many studies have shown that 5-HT regulates behavior and emotions and suppresses aggressive behavior caused by exposure to new environments [50]. The serotoninergic system plays an important role in anxiety-related behaviors [51]. Our results also demonstrate that 5-HT levels decreased in the fear circuit regions including PFC and HIP in SPS-exposed rats. However, MYR administration restored to normal 5-HT levels in the PFC and HIP. This suggests that MYR administration can modulate the 5-HT imbalance, which is a known pathophysiological mechanism of PTSD.

BDNF plays an important regulatory role in synaptic function and plasticity within specific circuitry of the HIP in the context of anxiety-like behaviors. Its expression was found to be decreased in the HIP of PTSD patients [34]. Therefore, we suggest that the functional disruption of the HIP induced by reduced BDNF expression may be closely related to anxiety-like symptoms [52]. MYR administration significantly reversed the SPS-induced reduction of BDNF mRNA expression, which suggests that its beneficial effects on depression- and anxiety-like behaviors were mediated by an increase in BDNF expression that may be associated with enhanced neuronal function.

BDNF reduction in animal models of PTSD augmented the response to traumatic stress and affected hippocampal function [53]. BDNF signaling is mediated by TrkB receptor activation, and phosphorylation of ERK protein could enhance contextual fear memory in PTSD [16, 54]. Therefore, modulation of the BDNF-ERK signaling pathway may increase fear-related freezing behavior and anxiety-like symptoms by enhancing hippocampal-dependent memory and promoting memory-related synaptic changes, as seen in long-term potentiation, for example [16, 54]. In our study, SPS-exposed rats exhibited decreased BDNF and TrkB mRNA expression and ERK phosphorylation in the HIP, but MYR administration reversed these reductions. The restoration of BDNF improved fear extinction and anxiety-like symptoms [54]. The antidepressant and anxiolytic effects of MYR may also be related to suppression of the ERK phosphorylation via modulation of BDNF levels. Our results show that MYR administration alleviated depression- and anxiety-like behaviors by regulating the BDNF-ERK signaling pathway.

MYR exerted antidepressant and anxiolytic effects in the FCT, FST, and EPM test, possibly by regulating the HPA axis and monoamines and activating the BDNF-ERK signaling pathway in our animal model of SPS. However, further studies are required to elucidate how MYR influences cell signaling pathways.

## 5. Conclusion

MYR is a potential therapeutic agent for fear memory, depression, and anxiety-like disorders caused by PTSD. MYR appeared to prevent monoamine imbalance through HPA axis regulation and activation of the BDNF-ERK signaling pathway.

## Figures and Tables

**Figure 1:** Experimental protocols for single prolonged stress (SPS)-induced anxiety-like behaviors and myricetin (MYR) treatment in rats. Different groups of rats (*n* = 8 per groups) were used for each experimental condition.

**Figure 2:** Results of body weight and sucrose intake analyses of rats subjected to 14 days of a SPS. Body weights and sucrose intake were significantly lower in SPS-exposed rats than in SAL-treated rats (significant main effect of SPS exposure *vs*. control handling). Data are shown as means ± standard errors of the mean. ^*∗∗*^*p* < 0.01 and ^*∗∗∗*^*p* < 0.001 *vs*. SAL group.

**Figure 3:** Effect of MYR on freezing behavior in response to conditioning (C1∼C3), extinction (E1∼E6), and short-term recall (R1) (a) and the percentage of time spent frozen during short-term recall (b) in the fear conditioning test, the immobility time (c), climbing behavior (d), and swimming time (e) in the forced swimming test (FST), the percentage of time spent in the open (f) and closed (g) arms, number of entries into the open (h) and closed (i) arms, and anxiety index (j) in the elevated plus maze (EPM) test after exposure to SPS in rats. ^*∗∗*^*p* < 0.01 and ^*∗∗∗*^*p* < 0.001 *vs*. SAL group; ^#^*p* < 0.05 and ^##^*p* < 0.01 *vs*. SPS group.

**Figure 4:** Effect of MYR on corticosterone (CORT (a)), adrenocorticotropic hormone (ACTH (b)), and corticotropin-releasing hormone corticosterone (CRH (c)) levels in the plasma and norepinephrine (NE) concentrations in the medial prefrontal cortex (d), hippocampus (e), and amygdala (f), and serotonin (5-HT) concentrations in the medial prefrontal cortex (g), hippocampus (h), and amygdala (i) of rats exposed to SPS for 14 days are shown. ^*∗*^*p* < 0.05 and ^*∗∗*^*p* < 0.01 *vs*. SAL group; ^#^*p* < 0.05 *vs*. SPS group.

**Figure 5:** Effect of MYR on the mean number of brain-derived neurotrophic factor (BDNF)-stained hippocampal areas in rats with SPS-induced depression- and anxiety-like behaviors. Representative photographs and the relative percentage values are indicated. ^*∗*^*p* < 0.05 *vs*. SAL group; ^#^*p* < 0.05 *vs*. SPS group.

**Figure 6:** Effect of MYR on the expression levels of brain-derived neurotrophic factor (BDNF) and tropomyosin-related kinase B (TrkB) mRNAs in rats hippocampal with SPS-induced depression- and anxiety-like behaviors (a). The relative intensities of polymerase chain reaction amplification product bands on agarose gels are shown. The expression levels of BDNF and TrkB mRNAs were normalized to the expression level of glyceraldehyde 3-phosphate dehydrogenase mRNA as an internal control. Activation of phosphor-extracellular signal-regulated kinase (p-ERK) in the hippocampus after MYR treatment (b). Western blot analysis of protein expression levels of p-ERK. ^∗^*p*<0.05 and ^∗∗^*p*<0.01 vs. SAL group; ^#^p<0.05 vs. SPS group.

## Data Availability

All data supporting the conclusions of this article are included within the article. The datasets used or analyzed during the current study are available from the corresponding author on reasonable request.
